The article "Chemical Composition, Pharmacological, and Toxicological Effects of Betel Nut" was retracted in 2023. Reasons: signs of a paper mill; compromised peer review; unreliable results or conclusions.

# Chemical Composition, Pharmacological, and Toxicological Effects of Betel Nut

**DOI:** 10.1155/2021/1808081

**Published:** 2021-08-18

**Authors:** Xiaoxiao Chen, Yongzhi He, Yanru Deng

**Affiliations:** ^1^College of Pharmaceutical Engineering of Traditional Chinese Medicine, Tianjin University of Traditional Chinese Medicine, Tianjin 301617, China; ^2^College of Traditional Chinese Medicine, Tianjin University of Traditional Chinese Medicine, Tianjin 301617, China

## Abstract

Betel nut, the fruit of *Areca catechu* L, has a long medical history in Southeast Asia. It is native to Malaysia and is cultivated and processed extensively in subtropical regions, such as South China and India. Betel nut almost appears as a “snack” in various occasions in most parts of China. Clinically, betel nut can play a certain pharmacology role and was used in malaria, ascariasis, arthritis, enterozoic abdominalgia, stagnation of food, diarrhea, edema, and beriberi. The nervous excitement of betel nut chewing has made it gradually become popular. However, chewing betel nut can induce oral submucosal fibrosis (OSF) and oral cancer (OC). At the same time, long-term chewing of betel nut also causes inhaled asthma, sperm reducing, betel quid dependence (BQD), and uterine and esophageal cancers. The main components of processed betel nut are the goal of this review. This study will mainly start from the pharmacological activity and toxicology study of betel nut in recent years, aiming to seek its advantages and disadvantages. In the meantime, this study will analyze and emphasize that betel nut and arecoline are the high-risk factors for oral cancer, which should arouse attention and vigilance of the public.

## 1. Introduction

Betel nut is the dried seed of the fruit from the *Areca* palm, which is cultivated particularly in South and Southeast Asian countries. According to the statistics, India, Malaysia, and Bangladesh have the world's largest annual production in the world. Meanwhile, betel nut is an important traditional Chinese medicine (TCM), which has been used since antiquity [1]. It is estimated [2] that about more than 600 million people chew and eat betel nut. In addition to its medicinal use, there is a widespread abuse of addiction of betel nut, which is considered the fourth most used stimulant.

## 2. Chemical Composition

So far, a variety of chemicals have been identified from betel nut, including alkaloids, tannins, flavonoids, triterpenoids, steroids, and fatty acids [3].

### 2.1. Alkaloids

The alkaloids in betel nut are the main active ingredients in research currently, while arecoline (methyl 1-methyl-3,6-dihydro-2H-pyridine-5-carboxylate) is considered the most important alkaloid in betel nut. It is the main active ingredient and also the major toxic compound. The total alkaloid content of betel nut is estimated between 0.3% and 0.7%. The alkaloids also include arecaidine, arecoline, arecolidine, guvacoline, guvacine, arecatannin A1, arecatannin A2, isoguvacine, homoarecoline, nicotine, and dichroine [4]. Recently [5], there are two new alkaloids, acatechu A and acatechu B (as shown in Figure 1), which are separated from betel nut and obtained their structures, and the study of the component in betel nut like alkaloids is still deepening.

The article "Chemical Composition, Pharmacological, and Toxicological Effects of Betel Nut" was retracted in 2023. Reasons: signs of a paper mill; compromised peer review; unreliable results or conclusions.

Arecoline is a pyridine-type alkaloid which can quickly cross the blood-brain barrier and that depends on its chemical structure [6], which lacks quaternary ammonium ions compared with methacholine and has higher lipophilicity, so it can cross the cell membrane into the body better. In each period of betel nut from young fruit to mature and then to processing and placement, the content of arecoline changed accordingly. The general trend is that the content will decrease after the peak of ripeness [7].

### 2.2. Tannins

Tannin is the major component which makes betel nut bitter and astringent. Proanthocyanidins are the main tannin component of betel nut, including catechins, arecatannin, and proanthocyanidin A and B [8, 9].

### 2.3. Flavonoids

Flavonoids [9], with various biological activities such as antibacterial and antitumor, are also isolated from betel nut. The main classes of flavonoids in betel nut are isorhamnetin, chrysoeriol, luteolin, quercetin, glycyrrhizin, jacareubin, flavan-3-ol, flavan-3,4-diols, 4′,5-dihydroxyl-3′,5′,7-trimethoxyflavone, and 5,7,4′-trihydroxy-3′,5′-dimethoxydihydroflavone [10, 11].

### 2.4. Triterpenoids and Steroids

Betel nut also contains triterpenoids compounds, including isotic acid and its derivatives and 3*β*-acetylursolic acid in betel nut, as well as aromatic alcohol, aromatic methyl ether, fernenol, aroin, cyclic altonil, and cycloartenol [12]. He et al. extracted arborinol, fernenol, and arundoin from betel nut [13]. The steroidal compounds are *β*-sitosterol, cycloartenol, stigmata-4-en-3-one, and 22-dien-3-ol [9].

### 2.5. Fatty Acids

It is normal to use supercritical fluid extraction (SFE) to distill fatty acids and use GC/MS to analyze volatile components in betel nut [14]. According to the study, there are lauric acid, nutmeg acid, palmitic acid, stearic acid, oleic acid, hexadanic acid, and (E,E)-2,4-decadienaldehyde from the betel nut peel [15].

### 2.6. Other Chemical Compounds

Studies of the betel nut composition yet contain multiple categories of compounds, for instance, He et al. [13] found chrysophanic acid and physcione. The polysaccharide in the betel nut is about 18.7%, mainly galactose and sucrose, and plays a main antioxidant role in betel nut. Besides, resveratrol [16], erulaic acid, ferulic acid, hervanonic acid, and deoxymethyl-iodinated lutein acrylic acid were also isolated from betel nut seeds.  Table 1 shows that the ingredients of betel nut.

The article "Chemical Composition, Pharmacological, and Toxicological Effects of Betel Nut" was retracted in 2023. Reasons: signs of a paper mill; compromised peer review; unreliable results or conclusions.

## 3. Pharmacological Effects

### 3.1. Digestive System Effects

Salehi and his colleagues [18] summarized the digestive system effects of betel nut, for example, insect repellents, digestive function enhancers, treatment of diarrhea, constipation, antiheartburn, ulcers, and dyspepsia, and also treat gastrointestinal inflammation, flatulence, hyperemesis gravida, and so on. It has been confirmed that arecoline can stimulate the sympathetic nerve, stimulate the choline *M* receptor, promote the increase of human saliva secretion, sweating, and excitement and gastrointestinal peristalsis, and help to improve human digestive function [19].

### 3.2. Antiparasitic and Antibacterial Effects

Some of the examples are antimalaria, treatment of leprosy, and antibacteria. Chusri et al. [20] investigated the biological activity of traditional herbal formulas to heal wounds and found that ethanol extracts containing betel nut and other four herbs can play an antibacterial role including against *Staphylococcus aureus* (SA), methicillin-resistant *Staphylococcus aureus* (MRSA), and so on. It also has significant antioxidant capacity for scavenging hydroxyl-free radicals.

In addition, Wang et al. [21] studied the anticoccidial effects of *Areca* nut extract (ANE) on coccidiosis, which showed that ANE could make the food consumption of rats and the mucosal damage improved. It explains that the betel nut has a certain extent anticoccidial activity and beneficial effect on tissue damage caused by coccidiosis.

### 3.3. Nervous System Effects

Betel nut can act on the nervous system and has the effects of antiaging, improving learning and memory. Arecoline has an acetylcholine-like effect, which can activate *M* receptors, thus stimulating the parasympathetic nerves. At the same time, arecoline also has an inhibitory effect on gamma-aminobutyric acid (GABA), which can bring delight and excitement. After arecoline enters the oral cavity, it will have a mild systemic choline effect [22]. Ono et al. [23] established an AD model in aged rats and gave them 10 mg/kg arecoline for 6 consecutive days. Experimental results found that this can improve the cognitive performance of elderly rats, which shows that arecoline has a certain pharmacological activity in improving some symptoms of Alzheimer's disease (AD). Furthermore, the research results of Asthana [24] showed that arecoline has a certain pharmacological effect on enhancing the memory of AD patients.

The article "Chemical Composition, Pharmacological, and Toxicological Effects of Betel Nut" was retracted in 2023. Reasons: signs of a paper mill; compromised peer review; unreliable results or conclusions.

### 3.4. Cardiovascular Effects

It can be used as an antihypertensive and diuretic. Some studies believe that betel nut is an herbal medicine with antihypertensive and blood lipid-lowering activities. Chewing betel nut will cause accelerated heartbeat, temperature rising, and heavy sweating within a certain period of time, promoting blood circulation. The research of Inokuchi [25] is suggested that the extract of betel nut has good hypotensive activity.

### 3.5. Other Effects

Some researchers have begun to study the active ingredients in betel nut that inhibit *α*-glucosidase [26]. Arecoline is considered a natural *α*-glucosidase inhibitor to treat postprandial hyperglycemia in diabetic patients. In vitro analysis, Nouri et al. [27] confirmed that the extract of betel leaves with different dissolvents can provide inhibitory effects on key enzymes (*α*-amylase and *α*-glucosidase) associated with type 2 diabetes and hyperglycemia. This allows us to determine that betel nut polyphenol has the pharmacological activity of lowering blood sugar, and it is based on the assumption that it plays a role in lowering blood sugar by inhibiting the activity of *α*-glucosidase.

Lee [28] found that arecoline (50 *μ*g/mL) can promote the survival and growth of glial cells in vitro and found that arecoline in the body can stimulate local inflammation, which can promote the repair of severe peripheral nerve damage.

In addition, it can also treat beriberi, low back pain [29], and remove bad breath. It also includes the effects of controlling sweating, edema, curing jaundice, and sedative effects [18].

## 4. Toxicological Effects

### 4.1. Bronchoconstriction

In vitro trials, arecoline is known to stimulate parasympathetic nerves and cause bronchial smooth muscle contraction, which is equivalent to a tenth of acetylmethylcholine. Taylor et al. [30] found that in the double-blind trial, subjects who chewed betel nut had bronchocontraction in different degrees. In the trials of four Bangladeshis asthmatic patients (AAPs) that chew betel nut regularly, there was one showing FEV1 that decreased 30% with symptoms of chest tightness within 150 minutes of chewing. It is speculated that betel nut contains arecoline, which acts as cholinergic alkaloids that stimulates the dose-related bronchocontraction.

### 4.2. Central Nervous Toxicity and Addiction

Adriane [31] found that when the neuroleptic drugs combine with betel nut, the extra propyramidal effect will be aggravated, and the combination of betel nut with trifluorothiotons and propylene cycling can cause stiffness, mild dyskinesia, and mandibular tremor. Combination with fluorosis can cause tremor, stiffness, and sensory abnormalities, and combination with prednisone and salbutiamine can cause asthma.

The article "Chemical Composition, Pharmacological, and Toxicological Effects of Betel Nut" was retracted in 2023. Reasons: signs of a paper mill; compromised peer review; unreliable results or conclusions.

Arecoline, a potentially addictive component of betel nut, is an oxidative inhibitor that suppresses monoamine oxidase A(MAO-A). Thus, it can prevent the decomposition of neurotransmitters, increasing the concentration of dopamine and serotonin in the brain, thereby bringing euphoria and happiness [32].Consequently, many betel nut chewers occur withdrawal symptoms after a long-term consumption of betel nut, which is as difficult to quit completely as tobacco. Withdrawal syndrome is characterized by mood swings, anxiety, irritation, inattention, sleep disorders, and increased appetite. According to the statistics, there are a large number of betel nut consumers around the world which has the betel quid dependence (BQD). Winstock et al. [33] reported that part of the subjects had a withdrawal reaction after stopping the betel nut chewing, with an average dependence severity of 7.3. Ko et al. [34] concluded by a systematic review that the neurological and pharmacological mechanisms behind BQD may be related to brain's reward, cognitive and impulsive system interconnection. Arecoline increases the level of brain serotonin and norepinephrine, showing that it can prevent the decomposition of neurotransmitters and improve dopamine (DA) and 5-HT levels in the brain.

### 4.3. Reproductive Toxicity

Recently, Wu [35] found that betel nut and arecoline had reproductive toxicity on male rats, including the decline of sperm amount, azoospermatism, and sperm morphological abnormalities, which lead to sperm function impaired. There is possibility that the extract of betel nut disturbs the sperm and human male reproductive ability. Yuan [36] reported that betel nut extract reduced the effect on human sperm motility, of which the effect of arecoline is the most remarkable. Another study [37] showed that the ethanol extract of betel nut had an effect on the weight of ovaries of female rats, which significantly increased the possibility of abortion. In general, betel nut contains components that may lead to human reproductive toxicity.

### 4.4. Cytotoxicity and Genotoxicity

Lin et al. [38] confirmed the effects of arecoline on the epigenome and evaluated the mRNA expression of histone methyltransferase, acetyltransferase, and demethylase in K-562 cells exposed to arecoline. In fact, arecoline makes the expression of related genes (M) that catalyze histone methylation, acetylation, and demethylation is altered. While, H3K9 methylation involves maintaining the stability of chromosomal structural and inactivation of autosomal gene expression. Available data indicate that arecoline-induced epigenic changes play a part in chemically mediated mechanisms of cytotoxicity and genotoxicity. Arecoline can induce DNA chain disruption, chromosome distortion, and sister chromatid exchange, affect DNA repair, and cause oxidative stress, and its metabolites, arecaidine and arecoline-N-oxide, are also genetically toxic [39] (Table 2).

The article "Chemical Composition, Pharmacological, and Toxicological Effects of Betel Nut" was retracted in 2023. Reasons: signs of a paper mill; compromised peer review; unreliable results or conclusions.

Shih's [40] study on the cytotoxicity of arecoline showed that arecoline increases cytochrome C release and activates the cysteine aspartate-specific protease related signaling pathway, inducing neuronal cell death. Inhibition of cell proliferation after arecoline addition may be caused by cell death induced by cytotoxicity of arecoline. In addition, Yen et al. [41] found that arecoline can inhibit AMPK, the AMP-dependent protein kinase, through inducing intracellular reactive oxygen substances, and it is responsible for performing cell apoptosis.

### 4.5. Carcinogenicity

Arecoline, an important ingredient in betel nut, has been regarded as a possible carcinogen for human beings by the International Cancer Research Institute [42]. IARC set betel nut as “Group2Bcarcinogens,” which means “may be carcinogenic to humans.” It was also observed that arecoline increased the incidence of tumors, such as inducing malignant tumors of the esophagus and tongue in animal experiments [39].

#### 4.5.1. Oral Carcinogenesis

In recent years, an increasing amount of data indicate that the habit of betel nut chewing is harmful to human oral health, even caused oral cancer, resulting in death or severe facial distortion [43] (as shown in Figure 2). It has been shown that the appearance of oral cancer is closely related to unhealthy oral habits, including betel nut chewing [44]. There are a series of studies that have found that oral cancer is due to carcinogenic agents such as arecoline, active oxygen, and nitrosamines, which are highly related to human toxicology [45]. In experiments on the interaction between those of are coline and human fibroblasts, the researchers confirmed that alkaloids of betel nut stimulate collagen synthesis, of which the effects of arecaidine are remarkable and in a concentration-dependent manner.

Chewing betel nut can induce oral leukoplakia and oral submucosal fibrosis (OSF), while OSF is an oral cancer (OC) precancerous state. Currently, Murti et al. [46] considered that the consumption of betel nut is the remarkable cause of OSF through ecological observations and case reports. The habit of chewing betel nut may cause oral precancerous lesions such as OSF with the possibility of malignant transformation [47]. When arecoline was administered in drinking water to GPT delta rats, the frequency of oral tissue mutations which were detected is at 2.5 times that of the untreated, showing a unique mutation spectrum. It is suggested that arecoline produces mutationally induced damage in the oral tissues of rats [48]. Moreover, N-nitrogenous derivatives of arecoline are a significant carcinogenic factor, which tends to oral squamous hyperplasia in mice [49]. Wang et al. [50] examined the RT-PCR and found that after removing HIF1A-AS1 gene segment, the arecoline-stimulated migration capacity in buccal mucosal fibroblasts (BMFs) was obstructed. Their results showed that arecoline may result to relatively overexpress in OSF tissues compared to normal tissue counterparts and can activate BMFs, which may be one of the pathogenic pathways of OSF. Lin et al. [51] found that OSF associated with chewing betel nut increases the chance of multiple oral cancers greatly. It is vital to prevent OSF and stop chewing betel nut for reducing the morbidity of OC. A recent meta-analysis of Yang et al. [52] found that the prognosis of patients with betel nut chewing habits was poorer than those not. Therefore, long-term betel nut users should be aware of the potential risk of cancer.

The article "Chemical Composition, Pharmacological, and Toxicological Effects of Betel Nut" was retracted in 2023. Reasons: signs of a paper mill; compromised peer review; unreliable results or conclusions.

#### 4.5.2. Risk of Other Cancers

Besides oral cancer that attracts public attention, arecoline may also be a contributing factor to esophageal, liver, lung, and other diseases. For example, Wu et al. [53] explored the association between chewing betel nut with liver cirrhosis (LC) and hepatocellular cancer (HCC). It was remarkable that betel nut caused the risk of LC and HCC increased by 4.25 times among subjects that still chew betel nut and caused the risk of infection with hepatitis B or hepatitis C. In fact, betel quid chewing has an increased synergistic effect on the risks associated with hepatitis B and hepatitis C, yet stopping chewing BQ can reduce the immune risk caused by hepatitis C. Hence, it might be said that chewing betel nut will induce liver cirrhosis and hepatocellular cancer. According to reports [54], there is an association between betel nut chewing and esophageal cancer, which can significantly increase the risk of cancers.

### 4.6. Nephrotoxicity

Wang et al. [55] researched many chronic kidney disease (CKD) patients and non-CKD patients and analyzed the effect of betel nut chewing on nephropathy. It showed that the betel chewer had a higher risk of CKD than others, which can speculate that chewing betel nut has nephrotoxicity and associated with CKD occurrence.

## 5. Conclusion

Through a series of studies, this review summarized the chemical composition of betel nut and pharmacology and research progress in clinical application of betel nut. Edible betel nut is more toxic, staying longer in the mouth, and using it for a long time is more likely to cause dependence than medicinal betel nut. The medicinal betel nut is generally weak in toxicity, with a small dosage and little harm to the human body. The difference between the two is mainly in the way of use. As one of the most effective components of betel nut, arecoline has pharmacological activities such as antibacterial and anthelmintic effects, reducing postprandial hyperglycemia and improving Alzheimer's disease. However, the harmful and side effects of betel nut cannot be ignored, including cytotoxicity and genetic toxicity, carcinogenicity (especially oral cancer), OSF, and addiction dependence. There are still a large number of people who are diagnosed with oral cancer, which is related to betel quid dependence (BQD) in consumers and improper promotion and guidance of enterprise. After clarifying the toxicology mechanism and potential risks of arecoline, the public should try to stay away from these substances.

The article "Chemical Composition, Pharmacological, and Toxicological Effects of Betel Nut" was retracted in 2023. Reasons: signs of a paper mill; compromised peer review; unreliable results or conclusions.

It is necessary to develop adjuvant therapeutic drugs for betel nut withdrawal syndrome of potential BQD cessation drugs. In areas like Taiwan, such dependence quit institutions have emerged. Furthermore, chewing betel nut is not the only carcinogenic factor; thus, the use of products, like electronic cigarettes, containing arecoline should also be eliminated. In conclusion, the proportion of betel nut as chewing snacks should be depressed gradually. The increased investment in research of betel nut effects is vital for future work, and betel nut will play a more positive role in pharmacological and medical fields through guidance and supervision rather than becoming an unregulated addictive substance.

## Figures and Tables

**Figure 1:** Chemical structures of acatechu A and B.

**Figure 2:** Oral diseases associated with betel nut.

**Table 1:** Ingredients of betel nut [17].

Classification	Ingredient name
Alkaloids	Arecaidine
	Arecaine
	Arecatannin a1
	Arecatannin a2
	Arecolidine
	Arecoline
	Arecoline
	4-Quinazolone
	*α-*Dichroine
	*β*-Dichroine
	Guvacine
	Guvacoline
	Homoarecoline
	Isoguvacine
	Methyl N-methylpiperidine-3-carboxylate
	Ethyl N-methylpiperidine-3-carboxylate
	Ethyl nicotinate
	Nicotine

Flavonoids	Isorhamnetin
	Chrysoeriol
	Luteolin
	Quercetin
	Glycyrrhizin
	Jacareubin
	4-Hydroxyhydrangenol

Tannins	(+)-Catechin
	Procyanidin A1, B1, B2, B3
	Arecatannin A1, A2, A3
	Arecatannin B1, B2
	Arecatannin C1

Terpenoids	3-Carene
	Procurcumenol
	Ursonic acid
	3-Acetylursolic acid,
	Arborinol
	Arborinol methyl ether
	Fernenol
	Arundoin

Steroids	Cycloartenol
	5, 8-Epidioxiergosta-6
	Beta-sitosterol
	22-Dien-3-ol
	Stigmasta-4-en-3-one

Fatty acids	2-Lauroleic acid
	Arachidic acid
	Cis-4-dodecenoic acid
	Cis-9, cis-12-linoleic acid
	Myristic acid
	Oleic acid
	Palmitic acid

Others	Vanillin
	Alpha-terpineol
	Benzyl alcohol
	Capric acid
	Caproic acid
	Resveratrol
	Quinic acid
	Dicoumarin

The article "Chemical Composition, Pharmacological, and Toxicological Effects of Betel Nut" was retracted in 2023. Reasons: signs of a paper mill; compromised peer review; unreliable results or conclusions.

**Table 2:** Summary of DNA damage by arecoline and its metabolites [39], (+) for positive results and (–) for negative results.

Compound	DNA breaks	Unscheduled DNA synthesis
Arecoline	(+) Mice kidney cells	(+) Early spermatid stages of Swiss albino mice cells
	(+) Human oral cells	(+) Hep-2 cells
	(+) Hep-2 cells	(−) Human gingival keratinocytes
	(+) 293 cells	
	(−) Rat liver clone 9 cells	

Arecoline-N-oxide	(+) Rat liver clone 9 cells	
	(+) Human oral cells	
	(+) Immunodeficient NOD/SCID mice	

Arecaidine	(+) Human oral cells	

3-(N-Nitrosomethylamino) propionaldehyde	(+) Human oral cells	
